The article "Analysis on the Correspondence between Sustainable Social Service Design and Humanistic Aesthetic Design and Cognitive Psychological Utility" was published in 2022. Journal: J Environ Public Health.

# Analysis on the Correspondence between Sustainable Social Service Design and Humanistic Aesthetic Design and Cognitive Psychological Utility

**DOI:** 10.1155/2022/7309888

**Published:** 2022-07-20

**Authors:** Yang Yu, Jiaji Gao, Nagai Yukari

**Affiliations:** ^1^School of Art and Design, Dalian Polytechnic University, Dalian 116034, Liaoning, China; ^2^School of Knowledge Science, Japan Advanced Institute of Science and Technology, Nomi 923-1292, Ishikawa, Japan

## Abstract

In this era of gradual scarcity of resources, sustainable development has become an important issue for society. In this environment, the cultural, economic, and social environment has a decisive influence on sustainable development. This paper mainly starts with service design and humanistic aesthetics and introduces the sustainable design development theory into the design so that the design can better respond to the sustainable development strategy. We established the integration method of marketing and design, through the combination of humanistic art design and the cognitive psychological effect and the cognitive psychological effect of customers, advocating appropriate design and humanism in the information age, which not only improves the sustainable society but also enriches the service design system theory.

## 1. Introduction

The current society is an important period of turning to a sustainable society, and the environmental, economic, and social issues arising under its specific background undoubtedly make sustainable social services have greater responsibility [1]. However, in the case of sustainable social service design, the corresponding relationship between sustainable social service design, humanistic aesthetic design, and cognitive psychological utility still needs to be discussed in detail [2]. Under the current situation of rapid development of today's society, at present, service design in Asia is relatively few, this idea is mainly popular in Europe, and in particular, the UK will develop relatively better. It is necessary to reflect on the phenomenon of today's social service design. Service design is a design activity that effectively plans and organizes the people, infrastructure, communication, and materials involved in a service to improve the user experience and service quality, which can analyze the drawbacks that will arise from the lack of design ethics in today's society, and Gao Mei from Zhengzhou University of Light Industry points out the status and responsibility of useless design in changing the way of social development, so as to the emergence of the useless design stage is the inevitable trend of the development of sustainable social service design theory. Among them, “useless design” is a new design concept. Useless design refers to the design of discarded items, excess waste from the manufacturing process, outdated items, etc., through manufacturing or even handcrafting under the condition of environmental protection principles, to transform the second life of the object, promote environmental awareness of using less materials, and emphasize design to create sustainable. It advocates for more direct value for consumers, society, or the world and for the sustainability of design. Professor Liu Xin of Tsinghua University discusses the meaning of the useless design concept and points out the progressive significance of the useless design concept in the new era: more emphasis is placed on the importance of combining humanistic art design with cognitive and psychological utility; it reverses the ethics of today's design, advocates moderate design and humanity in the information age, pays attention to people's emotional needs, reshapes people's concept of happiness, creates more direct value for society, optimizes “useless” resources, and pays attention to the design of nonmaterial forms [3], while the biggest characteristic of sustainable social service design is the fairness, sustainability, and commonality as the three basic principles [4].

“Sustainable design” is different from the general design that outputs purely material products [5]. It integrates products and services to build sustainable solutions to meet the specific needs of consumers, replacing them with “results” and “benefits.” It is a strategic design activity with the ultimate goal of reducing the wastage of resources and environmental pollution and changing the quality of people's social life [6]. It can be seen that sustainable social service design occupies a very important position in our life [7].

In the theory of social service design, the pension service is an indispensable part of it. With the more and more serious national aging, the pension service also needs to be updated. Under the background of China's increasingly obvious aging, smart pension is an inevitable trend of China's pension development [8]. The shrinking social labor force and the substantial growth of the elderly population in the future will completely change China's pension structure [9] and become the driving force for the development of intelligent elderly care. At present, most of the research on smart old-age care centers on technical realization and social system [10]. How to use technology and design to improve the current chaotic old-age service resources, high cost of old-age care, low penetration rate, scattered smart applications, insufficient social resource support, and computer anxiety caused by the use of the Internet and smart products for the elderly, smart community old-age service system issues such as sustainable development, and provide directions for the research and development of smart old-age care. This paper introduces the concept of situational awareness, subdivides the key influencing factors in the elderly care situation, and makes the “wisdom” in smart elderly care truly play its role so that intelligence is not only reflected in the intelligence of equipment and the passive acceptance of the elderly. More attention should be paid to the old-age support for the elderly and the way to guide their behavior, and ultimately achieve the purpose of improving the quality of life and the way [11]. Situational awareness is based on the environment, dynamic, overall insight into the ability of security risk; is based on the security data, from the global perspective of security threat identification, analysis, response disposal of a way, and ultimately for decision and action; and is the security ability of the ground, and it provides certain security for the security of pension services.

The final design strategy is proposed based on user, service, social, and device contexts. We design practice through the application of design strategies to verify its effectiveness and ultimately optimize the user experience and system development of the smart community elderly care service App, in order to contribute to the design research in the field of smart elderly care in China [12]. The specific design strategy is shown in Table 1.

In the design strategy of elderly care services, the psychological problems of the elderly should also be focused on.

Psychological effects are more common psychological phenomena and laws in social life; it is the causal reaction or chain reaction that the behavior or role of a certain character or thing causes corresponding changes in other characters or things. Like anything, it has both positive and negative meanings. Therefore, correctly understanding, understanding, mastering, and utilizing the psychological effect play very important roles and significance in people's daily life and work. Cognitive psychological utility is mainly reflected in the “customer perceived value.”

Products used for consumption mainly refer to material commodities, spiritual and cultural commodities, various labor services, and other intangible and nonmaterial commodities. Features are associated with value, and product value should be analyzed under specific issues [13]. The value must be measured in conjunction with the specific environment, and the value in different environments should be very different.

## 2. State of the Art

Value thinking is a rational way of thinking to deeply understand the needs of products or consumers. Businesses grow by providing value to customers and gaining self-interest through their products [14]. Porter believes that a company's competitive advantage is ultimately derived from the value a company can create for customers. With the development of enterprise management theory, the competitive advantage of enterprises has shifted from product and technology as the core to the customer as the core, and the customer's satisfaction and loyalty are deeply studied. Robert F. Lauterborm tried to go beyond the 4P theory. 4P marketing theory is summed down to a combination of four basic strategies, namely, product (Product), price (Price), promotion (Promotion), and channel (Place). Since the English characters of these four words are P, plus strategy (Strategy), they are referred to as “4P.” He constructed the theory of integrated marketing communication and proposed “4C marketing,” as shown in Figure 1.

This theory emphasizes the primacy of customer satisfaction, reduces customer costs as much as possible, and takes into account the convenience of customers' purchasing behavior process, and the management of sales channels should be customer-centric. His theory attempts to emphasize the element theory of repositioning marketing from the customer's perspective, which is different from the 4P theory [15]. It emphasizes that enterprises should first put the pursuit of customer satisfaction in the first place, strive to reduce the purchase cost of customers, and then fully pay attention to the convenience of customers in the purchase process, rather than determine the sales channel strategy from the perspective of the enterprise, and finally, effective marketing communications should also be implemented with consumers at the center [16].

The higher the customer value of the enterprise services, the higher the satisfaction, and the stronger the competitiveness of the enterprise. Customer value can be evaluated from three aspects: economic value (the cost value invested in realizing the goal), physical value (the practical application function value obtained by the customer), and psychological value (the satisfaction of the customer's psychological value). Its core research is the difference between the benefits and the costs (purchasing costs and postpurchase costs) that customers get from purchasing goods. The subjective consideration of the customer's consumption process is based on perception, so the customer's perceived value affects the customer's consumption behavior to a large extent. Customer value is a trade-off between the buyer's perceived product performance and the total cost of purchase. Therefore, Zeithaml (V.A.) proposed customer perceived value (CPV). His theory revolves around customers (people) as the main body of marketing and believes that customers will subjectively pay for products and services when they obtain products and services [17]. The cost is weighed against the perceived benefit, and a series of evaluations and feedback are made. Therefore, the customer-perceived value theory points to the trade-off between the benefits that people perceive subjectively and the costs they pay when consuming or obtaining services, and to evaluate the overall utility of products or services [18]. It further guides the customer value problem to the customer's own decision making, thus making it clear that the external value organization problem should be explained from the perspective of the customer information center, as shown in Figure 2.

Over the years of development, it can be classified into three logical perspectives (as shown in Table 2): “trade-off” logic, “level” logic, and “dimension” logic. The trade-off logic interprets customer-perceived value as the contrast between what customers can perceive and what they can perceive; the value hierarchy distinguishes the relationship between internal and external customer values; the value dimension deconstructs the multiplicity of value characteristics [19], a classification method. These three logics are not exclusive, but complement each other and analyze customer value from different perspectives (relevant information is shown in Table 2).

At the level of theoretical sorting, which is shown in Table 3, this paper summarizes “customer perceived value” into three theoretical entry points: trade-off logic, hierarchical logic, and dimension logic, so as to deepen the specific principal content of customer perceived value, in order to understand the rational and irrational customers at the cognitive behavior level and provide the basis for decision making. Furthermore, this paper combines the psychological theories, behavioral theories, social, and cultural theories related to customer perception and other theoretical demonstrations to construct a design clue from value, meaning to specific information carrier [20]. At the level of research perspective, this paper emphasizes establishing the perspective of the overall value relationship between customers, designers, enterprises, and products, so as to grasp the accurate design direction. On the one hand, the research takes “achieving customer satisfaction” as the core of product design breakthrough, emphasizing the “attraction” factor for customers in the market, flow interacts. This way of thinking is to place product goals in the value network and design with the logic of customer service.

## 3. Missing Customer Value in Design Work

At the level of strategy analysis, based on the analysis of customer perceived value, this paper demonstrates the relationship, elements, and key operation links of strategies. The system construction includes an organic design strategy of four core work links of “value identification,” “value path,” “value creation,” and “value realization.” It is characterized by taking customer perceived value as the guide, taking customer value analysis as the starting point for value opportunity exploration, and combining with customer mental model as the basis, the designer's value coding, and customer decoding as the core creation process [21]. We design problem solving in the interaction of scenes. At the end of this paper, the author describes the design practice process based on the product design strategy of customer perceived value. Its focus is to integrate customer value opportunity mining and product form meaning construction to achieve product value breakthroughs.

One of the important reasons why product design innovation brings market risks to enterprises is the lack of in-depth understanding of “customer value.” Generally speaking, the aesthetic objects of design aesthetics include at least four levels: form aesthetics, functional aesthetics, technological aesthetics, and cultural aesthetics. In recent years, with the deepening of design culture and concepts, elements related to human care such as natural ecology, social ecology, and social culture have become more and more important, and aesthetics has gradually penetrated into all aspects of human culture. Humanistic aesthetic design means that the design is full of humanistic care.

## 4. Application and Strategy Analysis of Service Design Value Added and Cognitive Psychology

The inherent “needs are satisfied one by one” design thinking has been difficult to adapt to the current market characteristics in today's era, often resulting in a lack of product competitiveness. Therefore, it is urgent to establish a “value added” that starts from the customer's mind and actively creates market opportunities. *Design Thinking*. Different from the traditional single design method based on engineering management, aesthetics, ergonomics, or psychology, this paper establishes a multidisciplinary knowledge interdisciplinary research method that combines marketing and design and is verified by psychological experiments. The proposed product design strategy research oriented to “customer: perceived value” is precisely in the context of diverse social cultures, guided by the deep customer perceivable value purpose, and “value added” as the breakthrough point, so as to carry out product design. Process is a design strategy that emphasizes utility, process, and system.

### 4.1. Design Decisions

Cognitive psychology believes that sensation refers to the initial processes of perceiving and encoding environmental energy; perception (also translated as perception) is composed of meaning, relationship, context, judgment, past experience, and the result of the mental processes in which memory comes into play. Cognition is the process of mental activity that integrates, interprets, and assigns meaning to the information obtained by the sense organs. When the designer faces the design task, the external and internal constraints are transformed into specific information and memory labels that can be understood, and the long-term memory and knowledge of the designer are retrieved for analysis, integration, evaluation, and decision making. This specific information is influenced by the experience formed by the memory code, which in turn helps the designer make decisions and judgments. The design behavior of the product is the value encoding (Encode) in the open environment, and the process of consumption and use of the product is the user's understanding and decoding (Decode) of the product information, as shown in Figure 3. These works do not stop at the specific artifact design, but focus on the development of theoretical method models and design tools that are instructive for design decision making and innovation processes toolkit.

The design innovation of the intelligent creative industry involves the integration and innovation of a series of elements such as products, spaces, and services. In order to let the design practitioners in the industry systematically master the different aspects of product and service design, the design and R&D team have applied it from architecture, user insights, role research, design scope definition, and feasibility analysis, to prototype testing, conceptual solutions, and design ideas. Research methods and tools develop a design innovation tool package for the field of intelligent building assembly industry, helping designers in this field to build a whole industry chain and a full-use sustainable design innovation toolkit.

Empathy generally refers to the psychological empathy. That is, we put yourself in the shoes of other emotions and emotions of the cognitive perception, grasp, and understanding. Empathy can be divided into four dimensions: perspective taking, empathic concern, fantasy, and personal distress. Psychological empathy is the psychological basis for embodying “value resonance” and an important theoretical basis and method for design thinking. Value resonance is the synchronization of perception and emotion between the subject and the object of the design, forming a state of mutual understanding. Designers need to achieve this state in order to meet specific social and human needs in the design of artificial objects. Achieving this “resonance” requires designers to study several key elements: discerning object values; in-depth understanding of mental models; coding of specific design information; and meaning construction in specific scenarios. The key point of delivering user value is that the communication and perception of design information can be synchronized in the different contexts of users and designers.

#### 4.1.1. Case 1

Ford Motor Company, with the help of psychological empathy theory, designed and developed “aging simulation clothes” by integrating multidisciplinary experts such as geriatrics, materials science, design science, and behavioral science when designing FOCUS vehicles. Wearing this set of “simulation clothes,” designers can personally experience various difficulties encountered by the elderly in cognition, function, behavior, and psychology, and then help the design team to understand the needs of elderly users more comprehensively and design more inclusive FOCUS cars. Once the car was launched, it was favored by both the elderly and the young, achieved huge market success, and became a successful case of empathy theory in inclusive design practice.

#### 4.1.2. Case 2

Interdisciplinary design team jointly established by the British National Medical Service, the Royal College of Art, and Imperial College, through empathy experience, immersive research, tracking, shooting, and observation. The problem is analyzed. Designers work with first responders, observe, interview, and learn from first responders in the ambulance. With this immersive empathy research method (empathy) and codesign process (codesign), humanized design solutions are completed. The new protocol designs a central stretcher in such a way that clinicians have 360-degree access to patients for safer and more effective treatment. The interior design avoids nooks and crannies where dust could accumulate, and all equipment and consumables are secured to one side of the vehicle via a simple and well-designed “work wall” for ergonomically placed medical materials and tools. Emergency teams place modular treatment packs into the vehicle before each shift, containing all the materials needed for a specific job, such as dressings, intubation, airway and oxygen kits, burns, and maternity kits, for precision care. The study found that the newly designed ambulance had clear advantages in treatment efficiency and infection control. According to the forecast of the financial model, the new design can save the UK about 40 million pounds of financial investment in emergency treatment, showing the contribution of psychological empathy at the design strategy level.

### 4.2. Middle-Level Psychology Research and Application

The second level of psychology is the study of information processing. Cognitive psychology believes that human is an information processing system of “symbol manipulation,” which has six functions:

These functions of humans are close to those of computers, as can be seen in Figure 4. According to the theoretical assumptions of cognitive psychology, any system can exhibit intelligence if it can perform the above six functions. Therefore, these six functions also constitute the theoretical basis of artificial intelligence. Semiotics attempts to describe the mechanisms of perception and representation, and is one of the important theoretical frameworks for design psychology research and practice. Among them, perceptual meaning refers to understanding users' activities and needs, while representation refers to transferring users' needs to product attributes. Through visual product attributes and possession and use of products, users construct meaning interpretation codes in specific social contexts and form interpretations of symbols.

### 4.3. Behavioral Guidance

The product must closely link the visual form with the meaning that can be understood and used, so as to guide people to correct operational behavior. The functional effectiveness of user actions, that is, usability and ease of use, is fundamental criterion for product design. The product should adapt to the human mental model at all times, reducing errors and difficulty of action in use. Norman points out that a product's visual structure helps users evaluate how a product should be used through three clues: ease of use, functional visibility, constraints, and mapping.

The bottom layer of psychology is to study the physiological process of human beings, that is, the emotional experience generated by the neural response process. Norman analyzed people's emotional elements according to the instinct level, behavior level, and spiritual level. He emphasized the emotional applicability and experience of design, and positive user experience must satisfy users' desires and attract them in order to help companies improve their competitive effectiveness, as shown in Figure 5.

### 4.4. Emotional Intervention

Humanized design can actively intervene and reshape people's psychology and emotions. From a psychological perspective, Csikszentmihalyi and Rochberg-Halton distinguish three modes of interaction between people and things (intuition, emotion, and cognition) that are important for experience, self-perception, and the meaning-making of products. Cognitive models can assess the nature of user-artificial world interactions. Aesthetic experience, as a way of trading psychological cognition, is not limited to the artifact itself, but is considered to be an underlying factor in all user experiences. Emotional patterns of transactions between users and artefacts relate to the way psychic energy is conducted. The experience flow is stimulated by the intrinsic rewards of trading with artificial objects, which in turn leads to positive feedback in the user's psychology and helps to reshape self-awareness and emotions.

With a flexible and variable back wing design that can be closed or opened, the modular smart car seat is designed to create a ride experience that promotes the emotional exchange of adjacent occupants while maintaining individual occupant privacy. The dynamic wingspan of the “partner seat” maximizes the occupant's need for human interaction and privacy, and the exterior of the vehicle is designed as a “bubble” of smart glass, with the help of transparent OLEDs on the glass. The emotional information of each passenger is displayed inside.

With the help of experimental tests, oral records, semantic analysis, and other methods, the design team conducts sampling and comparative research on factors such as color psychology and auditory cognition of prisoners, and explores the positive correction effects of color and sound on criminal behavior and criminal psychology. Finally, through the integration of interaction design, color design, sound design, and other elements, the interactive product design and service experience for the psychological correction of prisoners are developed. In the specially designed correctional room in the prison, the prisoners can actively intervene and treat their negative criminal psychology by interacting with the device to help them return to society as soon as possible.

Affected children are still growing, and psychological cognition, socioemotional, and motor development are important to them. The design of the Dutch Children's Oncology Medical Center takes into account the physical and psychological growth needs of sick children, and adopts a large number of bright colors and game-based situational design specially designed for children to guide children's positive emotions, eliminate the fear of seeking medical treatment, and improve the quality of life. We give them a more positive therapeutic mindset.

According to statistics, nearly 80% of pediatric patients in hospitals need to take sedatives for MRI examinations. When Philips designed the children's MRI equipment and testing space, with the help of experience design and service design methods, the MRI machine was transformed into a children's experience situation of adventure stories, in which the patient played the protagonist. With the help of multimedia projection technology, the design team constructed different game scenarios, such as underwater exploration, on the outside of the machine and in the room, and created a story script for the technicians to guide the child patients into the story characters. Through the design, the children regard the medical examination, which has always been regarded as serious and terrifying, as a game, and actively cooperate with the medical examination procedure with a more active and pleasant attitude. With the help of this emotional experience design, the number of children taking sedatives dropped to 10%. The design of many children's hospitals not only solves children's fear of hospitals and the troubles of parents but also creates a cultural and artistic healing environment, which has played a positive role in promoting rehabilitation from the perspective of design psychology.

### 4.5. Value Association

The process of people accepting the meaning of information is the interpretation of the denotation and connotation information of man-made objects. In denotation, the product needs to convey information about its function and the content it represents; connotation refers to the dimension of aesthetic value, which conveys people's subjective impressions and emotions about the product. People like familiar things, and familiarity provides psychological pleasure and security. Associative design should pay attention to a mental model that conforms to the familiarity and intelligibility of a specific group in a cultural context, thereby increasing the user's perception dimension and the density of information and energy transmission. People interact with “real” felt products and their meanings through psychological cognition and associative processes, thereby shaping the user's experience.

## 5. Conclusion

To sum up, this article breaks through the traditional single design method based on engineering management, aesthetics, human-machine, or psychology, and establishes a multidisciplinary knowledge cross-type research that integrates marketing and design and is verified by psychological experiments. The proposed product design strategy research oriented to “customer perceived value” is precisely in the context of diverse social cultures, guided by the deep customer perceivable value purpose, and “value added” as the breakthrough point, so as to carry out the product design process. A design strategy emphasizes utility, process, and system, to explore the corresponding relationship between sustainable social service design, humanistic aesthetic design, and cognitive psychological utility.

## Figures and Tables

**Figure 1:** 4C marketing.

**Figure 2:** Explanation of peripheral value organization problems with customer information centers.

**Figure 3:** Sustainable design process.

**Figure 4:** The six functions of the “symbol operation” information processing system.

**Figure 5:** Research and application of bottom-level psychology.

**Table 1:** Design strategies.

Design strategy	For elderly care scenarios, we propose strategies based on user contexts, including progressive quality of life contexts to guide users' healthy and life, and integration of multiple contexts to provide users with personalized experience.
	Aiming at the improvement of the experience and adaptability of the elderly in the process of using the App, a strategy of intervening pension assistants to form three types of auxiliary modes based on social context is proposed, and a multi-user human-machine collaboration based on implicit interaction is proposed in the service context and working mode, including strategies for enhancing the perception ability of the elderly in the form of multisensory interaction in the context of equipment.
	We analyze the limitations and problems in the current pension model and pension service system, and propose strategies to improve users' perceived service quality based on service contexts, as well as strategies to enhance social participation in social contexts and make the system sustainable.

**Table 2:** Analysis of customer value from different angles.

“Trade-off” logic	“Level” logic	“Dimension” logic
The core of the trade-off logic is a comparison relationship. Think of customer value as a comparison is between total benefits and total costs for customers. It is believed that customers are always inclined to obtain more benefits from them, so as to obtain customer satisfaction. Analysis under this logic is often macroscopic, and at the same time, it is easy to ignore nonsubstantial and measurable content such as perceptual factors.	Hierarchical logic is based on customer needs and is gradually stratified from the core to the appearance based on the customer's value purpose. It regards the customer transaction process as a dynamic theory that is embedded in specific scenarios. He believes that customers' “expectation, perception, evaluation, and satisfaction” are based on their value goals. He goes beyond the category of the product itself and puts the customer into a behavioral process, combining the user”s experience in the context to understand the value connotation of the customer.	Dimension (or system) logic emphasizes different aspects of customer perceived value, deeply analyzes the specific perceived gains and losses of customers, and systematically subdivides customer value. This study allows researchers to distinguish between primary and secondary values and to identify the associated relationships. According to different dimensions of customer value, enterprises can adopt different innovative development strategies to meet specific customer needs in terms of product value. Because of the specific analysis of system logic, it will face a variety of possibilities, so there are many research cases under this logic, each with its own emphasis.

**Table 3:** Theoretical review.

Theoretical entry point	Theoretical argument
Logic of trade-offs	Psychological theory
Hierarchical logic	Behavioral theory
Dimensional logic	Sociocultural theory

## Data Availability

The labeled data set used to support the findings of this study is available from the corresponding author upon request.
